# The Role of Digital X-Ray in Curative Effect and Nursing Evaluation of Cervical Spondylotic Radiculopathy

**DOI:** 10.1155/2021/5666136

**Published:** 2021-08-16

**Authors:** Xue Chen, Pan Xue, Yuanyuan Shi, Si Chen

**Affiliations:** ^1^Department of Orthopedics, The Second Hospital of Jilin University, Changchun 130041, China; ^2^Department of Nursing, The Second Hospital of Jilin University, Changchun 130041, China; ^3^Geriatric Medicine, The Second Hospital of Jilin University, Changchun 130041, China

## Abstract

The present study attempted to analyze the features of atlanto-occipital radiograph in patients with cervical spondylotic radiculopathy or vertebral artery type. In order to reduce the interference of human factors and the measurement error as much as possible, this experiment adopts the blind design and analyzes the digital format X-ray films by using the computer software ImageJ. Because the tangent line between the outer plates of the anterior and posterior margin of the foramen magnum was not accurately located on the X-ray film, the angle formed by the line between the saddle dorsal slope and the center point of the anterior and posterior nodule with a clear display was selected as the measurement method of the angle between the atlanto-occipital joints. The results showed that the lateral cervical curvature of the VCS group was 0.43 ± 0.51, and the lateral cervical curvature of the CSR group was 0.46 ± 0.49, both of which were significantly lower than the normal value (1.2 ± 0.5 cm). Patients in both groups had the characteristic of cervical curvature straightening. The changes of cervical curvature in overflexion and overextension positions can indirectly reflect the state of cervical motion. The anterior flexion neck curve of the VCS group was less than that of the CSR group (*P* < 0.05). Compared with the CSR group, VCS showed limited cervical anterior flexion movement. In this study, X-ray films of both CSR and VCS showed occipitocervical flexion and extension disorders, cervical curvature straightening, and lower cervical instability. In VCS, occipitocervical flexion and extension disorders were mainly manifested in atlantoaxial flexion disorders, while in CSR, atlanto-occipitocervical flexion and extension disorders were mainly manifested in atlantoaxial flexion disorders.

## 1. Introduction

Cervical spondylosis is a common disease in orthopedic department. The prevalence rate of cervical spondylosis in China is about 3.8%∼17.5%, and it shows a rapid increase and younger trend. Cervical spondylotic radiculopathy accounted for more than 60% of all types of cervical spondylopathy. The rotation and lifting technique is an important TCM method to treat cervical spondylotic radiculopathy. The method has been approved by the National Tenth Five-Year Project, the National Eleventh Five-Year Support Plan, and the National Natural Science Foundation of China, has proved its effectiveness and safety, and has been approved by the State Administration of Traditional Chinese Medicine to promote and apply nationwide. However, the basic research on the mechanism of action of this technique has been lagging behind and cannot meet the clinical needs.

In the preliminary clinical study, it was found that the X-ray manifestations of cervical spondylotic radiculopathy may be different from those of other types of cervical spondylopathy. Reviewing the previous literature, it is found that the summary analysis on the imaging manifestations of cervical spondylopathy of nerve radiculopathy is more common, but the comparative studies on the imaging manifestations of cervical spondylopathy of nerve radiculopathy and other types of cervical spondylopathy are rarely carried out.

Cervical spondylosis is caused by a series of clinical manifestations caused by cervical intervertebral disc degeneration, intervertebral instability, osteophyte or disc rupture at the vertebral edge, pulposus prolapse, and other compression of nerve roots, spinal cord, or vertebral artery. Cervical spondylotic radiculopathy (CSR) and vertebral artery spondylopathy (VCS) are the most common types of cervical spondylopathy. Clinically, both of them have their own unique clinical manifestations. However, there is no consensus on whether there is the same difference in imaging between the two. With the development of science and technology, imaging diagnostic technology has been improved and developed, and CT and MRI examination has been basically the universal application. However, because it is cheap and easy to perform, X-ray examination is still the most commonly used examination method for cervical spondylosis. Reviewing the previous literature, the summary and analysis of X-ray films of cervical spondylosis are more common, but the comparative analysis of X-ray findings of cervical spondylosis of nerve root type and cervical spondylosis of vertebral artery type is rarely carried out. The analysis of the imaging findings of CSR and VCS is helpful to understand the pathogenesis of both and can improve the level of clinical diagnosis, which has important clinical value. Therefore, this experiment was designed to compare and analyze the X-ray characteristics of CSR and VCS.

Cervical spondylosis is caused by a series of clinical manifestations caused by cervical intervertebral disc degeneration, intervertebral instability, osteophyte or disc rupture at the vertebral edge, pulposus prolapse, and other compression of nerve roots, spinal cord, or vertebral artery. There are many research studies on the treatment of cervical spondylosis. The objective of this study was to investigate the curative effect of shock wave combined with acupuncture in the treatment of senile cervical spondylotic radiculopathy [1]. Zhou et al. studied the clinical efficacy of Baimai plaster massage combined with cervical pain granules in the treatment of cervical spondylotic radiculopathy [2]. Cui et al. discussed the efficacy of low-weight continuous traction in treating nocturnal pain of cervical spondylosis [3]. Juan et al. discussed the clinical efficacy of joint loosening combined with nerve loosening in the treatment of cervical spondylotic radiculopathy [4]. Sheng et al. discussed the clinical efficacy of acupuncture combined with cervical pain granules in treating cervical spondylotic radiculopathy [5]. Zhang et al. studied the clinical efficacy of warm acupuncture under the guidance of high-frequency ultrasound in the treatment of cervical spondylotic radiculopathy [6]. Jiang et al. discussed the application effect of TCM nursing clinical pathway in patients with cervical spondylotic radiculopathy [7]. Chen et al. analyzed the clinical efficacy of acupuncture, traction, and cervical vertebra in the treatment of cervical spondylotic radiculopathy [8]. Yang et al. analyzed the efficacy of Xifeng dredging collaterals combined with Shujing tongdu point in the treatment of vertebral artery type cervical spondylosis [9].

X-ray examination is the cheapest, is simple and easy to perform, and is often used in routine detection and diagnosis of cervical spondylosis [10]; it is a routine examination method for cervical spondylosis and has important clinical significance for the diagnosis of cervical spondylosis. It is generally believed that radiculotype cervical spondylopathy is mainly related to lower cervical spondylopathy and osteophyte hyperplasia, while vertebral artery type cervical spondylopathy is mainly manifested as atlantoaxial joint unalignment or cervical instability. In the previous literature, experimental designs were designed to summarize the X-ray manifestations of cervical spondylotic radiculopathy or vertebral artery spondylopathy without comparative analysis of the X-ray manifestations of the two. The difference in radiographic appearance between the two is inconclusive. There have been few studies on the findings of atlanto-occipital radiograph in patients with cervical spondylotic radiculopathy or vertebral artery type. Therefore, on this basis, this paper studied the curative effect of digital X-ray in cervical spondylotic radiculopathy. Cervical spondylotic radiculopathy is mainly manifested in atlanto-occipital joint extension disorder, while vertebral artery type cervical spondylopathy is mainly manifested in atlantoaxial joint flexion disorder, and this difference is closely related to its pathological mechanism.

## 2. Research Methods

### 2.1. Experiment Design: Single-Blind Control

#### 2.1.1. Sample Size

  Observation group: 60 cases of cervical spondylotic radiculopathy.
  Control group: 60 cases of vertebral artery type of cervical spondylosis.

### 2.2. Implementation Method

120 cases of X-ray films were randomly sorted, and then four clinicians trained in measurement were assigned to measure the numbered X-ray films without knowing the type of cervical spondylosis and input corresponding data. After data entry is completed, the analyst will break the blind and complete data statistical analysis.

### 2.3. Content and Method of Line Slice Measurement

The computer software ImageJ was used for imaging measurement. During measurement, X-ray film in DICOM format was imported into the program to open, and the drawing tool and measurement tool of ImageJ were used for measurement. Specific measurement contents and methods are as follows:

1. Cervical curvature: the distance between the posterior edge of the cervical curvature vertex vertebra and the tip edge of the axial odontoid process and the posterior lower edge of the seventh cervical vertebra was measured (curve convex is positive, and curve backward tensioning is negative).
2. Interangle: the angle formed along the saddle dorsal slope and the central point of the anteroposterior atlas nodules (positive angles are those located behind the cervical vertebra and negative angles are those located in front of the cervical vertebra) (see Figure 1).
3. C1/C2 angle: the angle between the line between the central point of the anterior and posterior atlas nodules and the tangent line of the lower margin of the C2 vertebral body (positive angle is located behind the cervical vertebra body, and negative angle is located in front of the cervical vertebra body).
4. C2/C3 angle: the degree formed by the tangent of the articular plane of the lower edge of the C2 vertebral body and the tangent of the lower edge of the C3 vertebral body (positive angle is located behind the cervical vertebra body, and negative angle is located in front of the cervical vertebra body).
5. Posterior spacing of C0/C1: the shortest distance between the occipital bone and the posterior atlas tubercle.
6. Posterior spacing of C1/C2: the shortest distance between the posterior atlas tubercle and the axial spinous process.
7. Lower cervical instability segment: on the cervical functional radiograph, angle >11° was formed between the vertebrae at the point where the extension line intersected the lower edge of the sliding vertebrae and the sum of the distance from the lower edge of the sliding vertebrae to the sum of the distance from the same vertebrae to the posterior edge of the same vertebrae ≥2 mm.
8. Interarticular angle flexion range: the difference between the interarticular angle on the anterior flexion film and the interarticular angle on the lateral film.
9. Extension range of motion of inter-articular angle: the difference between the inter-articular angle of the post extension film and the inter-articular angle of the lateral film.

## 3. Result Analysis and Discussion

### 3.1. X-Ray Analysis

#### 3.1.1. Cervical Curvature

Comparison of cervical curvature between the two groups is shown in Table 1.

#### 3.1.2. Angle between C0 and C1

Comparison of angle between C0 and C1 between the two groups is given in Table 2.

#### 3.1.3. Angle between C1 and C2

Comparison of C1 and C2 angles between the two groups is given in Table 3.

#### 3.1.4. Angle between C2 and C3

Comparison of C2 and C3 angles between the two groups is given in Table 4.

#### 3.1.5. C0/C1 Rear Spacing

Comparison of posterior spacing of C0/C1 between the two groups is given in Table 5.

#### 3.1.6. Back Spacing of C1/C2

Comparison of posterior spacing of C1/C2 between the two groups is given in Table 6.

#### 3.1.7. Correlation Analysis of Angular Flexion Change between C1 and C2 and Posterior Space Flexion Change

Correlation between anterior flexion of C1/C2 angle and posterior distance is given in Table 7.

#### 3.1.8. Lower Cervical Instability

Comparison of the proportion of lower cervical instability between the two groups is given in Table 8, and comparison of the distribution of lower cervical instability segments between the two groups is given in Table 9.

## 4. Discussion

The experimental results, as known from Table 1, show that the lateral cervical curvature of the VCS group was 0.43 ± 0.51 and the lateral cervical curvature of the CSR group was 0.46 ± 0.49, both of which were significantly lower than the normal value (1.2 ± 0.5 cm), as shown in Figure 2, suggesting that patients in both groups had the characteristics of cervical curvature straightening. When the cervical spine flexes forward, the cervical spine flexes and moves forward, causing the reduction of cervical curvature. The opposite is true for stretching. Therefore, the changes of cervical curvature in the overflexion and overextension positions can indirectly reflect the state of cervical motion. The anterior flexion neck curvature of the VCS group was less than that of the CSR group (*P* < 0.05), as shown in Figure 3, suggesting that the VCS had limited cervical anterior flexion movement compared with the CSR group.

The occipital neck has a large range of flexion, extension, and rotation. The flexion and extension of the neck is mainly completed by the atlanto-occipital joint, which accounts for half of the whole range of neck motion. The left and right rotations of the head and neck are mainly completed by the atlantoaxial joint, and its motion range can also account for about half of the entire rotation of the neck. The normal range of flexion and extension of atlanto-occipital joint and atlantoaxial joint was ±13° and ±10°, respectively. In this experiment, from Tables 2–6, the range of flexion and extension of atlanto-occipital joint in both groups was significantly less than the normal range, suggesting that both groups had atlanto-occipital flexion and extension disorders. Among them, the atlanto occipital joint extension dysfunction of CSR is more serious than that of VCs (*P* < 0.01). The range of flexion and extension of the atlantoaxial joint in both groups was significantly less than the normal range, indicating the presence of atlantoaxial flexion and extension dysfunction in both groups. Among them, the atlantoaxial flexion dysfunction of VCS was more significant than that of CSR (*P* < 0.05).

Radical cervical spondylopathy (CSR) is caused by disc degeneration, herniation, segmental instability, hyperosteogenesis, or osteophyte formation that irritates and compacts the cervical nerve roots in the spinal canal or in the foraminal area. During cervical anterior flexion, the ligamentum flavum and the posterior longitudinal ligament were elongated, and the sagittal diameter of the cervical canal and the area of the intervertebral foramen were increased accordingly, which could relieve the mechanical compression of nerve roots. However, cervical posterior extension activity can cause contraction of posterior cervical muscle group and reduction of intervertebral foraminal area and further aggravate neck, shoulder, and arm pain by irritating the pathological segmental nerve roots. Therefore, in patients with CSR, posterior extension activity disorders in upper neck are particularly obvious, while anterior flexion activity disorders are less severe than VCS. The two major curves of the vertebral artery are located in the occipital atlantoaxial complex. According to the mechanical compression theory, excessive cervical spine movement can cause the spatial changes of the cervical structure, especially the spatial changes of the occipito-atlantoaxial complex, resulting in the insufficiency of blood supply to the vertebral artery and inducing dizziness. Therefore, upper cervical flexion and extension dysfunction in VCS patients is a state of self-preservation. Furthermore, the vertebral artery was bent almost at right angles above the upper mouth of the transverse foramen of the atlas and was fixed in the groove of the vertebral artery of the atlas by the posterior membrane of the atlas. During cervical anterior flexion, the posterior atlanto-occipital membrane is stretched and local tension is increased, thereby compacting the vertebral artery across the atlanto-vertebral artery sulcus, resulting in insufficient blood supply. Thus, atlanto-occipital flexion dysfunction was more pronounced in VCS patients than in CSR.

In the course of flexion and extension of occipito-atlantoaxial joint, the posterior distance of occipito-atlantoaxial joint and occipito occipital joint changed accordingly. Therefore, this experiment is an attempt to analyze and study this index. The experimental results are given in Table 7, and there was no significant difference between the two groups in the statistical analysis of the posterior space between the occipito-atlanto joints at all states, and no statistical results consistent with the occipito-atlanto angle were obtained. The consideration is related to the difficulty in determining the occipital condylar boundary. In the VCS group, the change value of flexion activity in the posterior space of the atlantoaxial joint was smaller than that in the CSR group (*P* < 0.05), suggesting that the flexion activity of the atlantoaxial joint was limited in the VCS patients, which was consistent with the statistical results of the atlantoaxial angle. There was a positive correlation between the atlantoaxial angle and the change of flexion activity in the distance behind the atlantoaxial joint (*R* = 0.622) (*P* < 0.001). Comparatively speaking, the posterior distance of atlantoaxial joint is easier to measure than the angle between atlantoaxial joints, so the former is recommended in clinical practice.

Lower cervical instability is one of the imaging diagnostic criteria for vertebral artery type of cervical spondylosis, but it is also common in other types of cervical spondylosis. The results of this experiment are given in Tables 8 and 9, and the incidence of lower cervical instability was 58.3% in the VCS group and 51.7% in the CSR group, and there was no statistical difference between the two groups. The distribution of lower cervical instability segments in both the CSR group and the VCS group was concentrated in C3, C4, and C5, which was consistent with previous literature. There was also no statistical difference in the distribution of lower cervical instability between the two groups. These results suggest that lower cervical instability is only a manifestation of cervical degeneration and is not the characteristic X-ray finding of vertebral artery or radiculotype cervical spondylosis.

In this study, X-ray films of both CSR and VCS showed occipitocervical flexion and extension disorders, cervical curvature straightening, and lower cervical instability. However, there were some differences in the X-ray findings between the two, among which the occipitocervical flexion and extension disorders in VCS were mainly manifested in atlantoaxial flexion disorders, while the CSR was mainly manifested in atlanto-occipitocervical flexion and extension disorders, and the differences were closely related to their respective pathological mechanisms. In this study, the open position and double oblique profile of CSR and VCS have not been compared and analyzed, and further study is needed.

## 5. Conclusions

Occipital and cervical flexion and extension disorders, cervical curvature straightening, and lower cervical instability are common X-ray manifestations of radiculotype cervical spondylopathy and vertebral artery type cervical spondylopathy.

Cervical spondylotic radiculopathy is mainly manifested in atlanto-occipital joint extension disorder, while vertebral artery type cervical spondylopathy is mainly manifested in atlantoaxial joint flexion disorder, and this difference is closely related to its pathological mechanism.

## Figures and Tables

**Figure 1:** Measurement method of upper cervical intervertebral angle and posterior space.

**Figure 2:** Comparison of cervical instability between the two groups.

**Figure 3:** Comparison of cervical instability segment distribution between the two groups.

**Table 1:** Comparison of cervical curvature between the two groups (unit: cm).

The neck piece	Group	Mean ± SD (cm)	*t*	*P*
Side a	VCS	0.43 ± 0.51	−0.313	0.755
	CSR	0.46 ± 0.49		

Top down	VCS	−0.62 ± 0.41	2.088	0.039^*∗*^
	CSR	−0.77 ± 0.37		

After sticking a	VCS	1.24 ± 0.55	0.403	0.688
	CSR	1.20 ± 0.51		

Flexion or value	VCS	1.83 ± 0.70	−1.138	0.257
	CSR	1.97 ± 0.60		

^*∗*^The curvature of the anterior flexion cervical spine in the VCS group was lower than that in the CSR group, with statistically significant difference (*P* < 0.05).

**Table 2:** Comparison of angle between C0 and C1 between the two groups (unit: angle).

	Group	Mean ± SD (cm)	*t*	*P*
Side a	VCS	57.50 ± 8.49	−0.340	0.735
	CSR	58.13 ± 10.35		

Top down	VCS	53.86 ± 9.84	0.032	0.974
	CSR	53.80 ± 9.42		

After sticking a	VCS	66.70 ± 9.59	1.435	0.154
	CSR	63.73 ± 11.49		

Before the degree	VCS	2.96 ± 5.23	−1.038	0.302
	CSR	4.12 ± 5.49		

After elongation	VCS	8.81 ± 5.93	2.927	0.004^*∗*^
	CSR	5.64 ± 5.10		

Flexion extension range	VCS	12.28 ± 6.10	1.780	0.078
	CSR	9.78 ± 7.17		

^*∗*^The extension range of motion between C0 and C1 angles in the VCS group was significantly larger than that in the CSR group. The difference was statistically significant (*P* < 0.01).

**Table 3:** Comparison of C1 and C2 angles between the two groups (unit: angle).

	Group	Mean ± SD (cm)	*t*	*P*
Side a	VCS	27.11 ± 4.76	−2.325	0.022^*∗*^
	CSR	29.40 ± 5.74		

Top down	VCS	20.98 ± 6.31	−0.979	0.330
	CSR	22.04 ± 5.43		

After sticking a	VCS	31.72 ± 5.66	−0.990	0.324
	CSR	32.74 ± 5.43		

Before the degree	VCS	5.94 ± 3.45	−2.045	0.043^#^
	CSR	7.35 ± 3.89		

After elongation	VCS	4.62 ± 4.21	1.840	0.068
	CSR	3.34 ± 3.22		

Flexion extension range	VCS	10.74 ± 4.79	−0.056	0.956
	CSR	10.69 ± 4.53		

^*∗*^Lateral C1/C2 angle in the VCS group was lower than that in the CSR group, with statistically significant difference (*P* < 0.05). ^#^The flexion range of C1/C2 angle in the VCS group was smaller than that in the CSR group (*P* < 0.05).

**Table 4:** Comparison of C2 and C3 angles between the two groups (unit: angle).

	Group	Mean ± SD (cm)	*t*	*P*
Side a	VCS	1.75 ± 4.27	−0.743	0.457
	CSR	2.47 ± 3.23		

Top down	VCS	−2.55 ± 4.40	−1.146	0.254
	CSR	−1.65 ± 4.06		

After sticking a	VCS	4.75 ± 4.94	0.762	0.448
	CSR	4.15 ± 3.42		

Before the degree	VCS	4.54 ± 3.72	0.619	0.537
	CSR	4.12 ± 3.49		

After elongation	VCS	2.72 ± 3.63	1.800	0.075
	CSR	1.68 ± 2.51		

Flexion extension range	VCS	7.30 ± 4.36	2.011	0.047
	CSR	5.80 ± 3.65		

There was no statistically significant difference in the angle between the two groups.

**Table 5:** Comparison of posterior spacing of C0/C1 between the two groups (unit: cm).

	Group	Mean ± SD (cm)	*T* or *Z*	*P*
Side a	VCS	0.57 ± 0.30	−0.065	0.948
	CSR	0.57 ± 0.28		

Before the degree	VCS	0.64 ± 0.30	−0.849	0.398
	CSR	0.68 ± 0.28		

After elongation	VCS	0.20 ± 0.23	0.165	0.869
	CSR	0.20 ± 0.22		

Forward bending change value	VCS	0.06 ± 0.23	−1.229	0.222
	CSR	0.11 ± 0.24		

Change in extension	VCS	0.38 ± 0.25	0.007	0.994
	CSR	0.28 ± 0.25		

Flexion or value	VCS	0.44 ± 0.28	−0.975	0.311
	CSR	0.49 ± 0.31		

There was no statistically significant difference in the posterior space between the two groups.

**Table 6:** Comparison of posterior spacing of C1/C2 between the two groups (unit: cm).

	Group	Mean ± SD (cm)	*T* or *Z*	*P*
Side a	VCS	0.48 ± 0.23	0.474	0.637
	CSR	0.46 ± 0.21		

Before the degree	VCS	0.74 ± 0.28	−1.051	0.296
	CSR	0.80 ± 0.28		

After elongation	VCS	0.31 ± 0.15	−0.673	0.503
	CSR	0.33 ± 0.15		

Forward bending change value	VCS	0.26 ± 0.16	−2.157	0.033^*∗*^
	CSR	0.33 ± 0.20		

Change in extension	VCS	0.17 ± 0.18	1.192	0.236
	CSR	0.14 ± 0.11		

Flexion or value	VCS	0.43 ± 0.22	−0.896	0.372
	CSR	0.47 ± 0.21		

^*∗*^The flexion change of C1/C2 posterior space in the VCS group was less than that in the CSR group, with statistically significant difference (*P* < 0.05).

**Table 7:** Correlation between anterior flexion of C1/C2 angle and posterior distance.

Indicators	Forward flexion variation of the posterior spacing of C1/C2
Forward flexion between C1 and C2 angles	0.622^*∗∗*^

^*∗∗*^*P* < 0.001 indicates a significant correlation between the two.

**Table 8:** Comparison of the proportion of lower cervical instability between the two groups.

	Instability	No instability	X2	*P*
VCS	35	25	0.539	0.463
CSR	31	29		

There was no statistically significant difference in the proportion of lower cervical instability between the two groups.

**Table 9:** Comparison of the distribution of lower cervical instability segments between the two groups.

The section of instability	VCS	CSR	X2	*P*
C3	9	9	0.133	0.936
C4	17	15		
C5	8	6		
C6	1	1		
C7	0	0		

There was no statistically significant difference in the distribution of lower cervical instability between the two groups.

## Data Availability

The data used to support the findings of this study are available from the corresponding author upon request.
